This article has been retracted.

# Predictive Analysis and Evaluation Model of Chronic Liver Disease Based on BP Neural Network with Improved Ant Colony Algorithm

**DOI:** 10.1155/2021/3927551

**Published:** 2021-11-15

**Authors:** Na Jiang, Zhiwei Zhao, Pan Xu

**Affiliations:** Department of Gastroenterology, Hankou Hospital, Wuhan 430012, Hube, China

## Abstract

Timely prediction of the mechanism and characteristics of chronic liver disease using next-generation information technology is an effective way to improve the diagnosis rate of chronic liver disease. In this paper, we have proposed a modified backpropagation (BP) neural network with improved ant colony optimization algorithm to process multiple index attribute items describing chronic liver disease and construct a chronic liver disease assessment model. The proposed model is very effective in detecting chronic liver disease on time with acceptable level of accuracy and precision ratio. To verify these claims, the proposed scheme is checked experimentally where 125 groups of 20-dimensional medical test index data items of patients with chronic liver disease were analyzed. Moreover, 13-dimensional index items were preferentially selected as test index attribute items with high sensitivity to chronic liver disease using well-known ROC curves. The 13-dimensional index items were reduced to 5-dimensional comprehensive data items by principal component analysis. The proposed neural network-based model was trained with 115 sets of test indicator sample sets, and the remaining 10 sets of sample sets were used as test samples. Compared with the original 20-dimensional data as the neural network input, the proposed model not only reduces the complexity but also improves the prediction accuracy by 15.07%.

## 1. Introduction

Throughout the world, approximately 400 million people suffer from chronic liver disease [1]. There are many types of chronic liver disease such as chronic hepatitis A, chronic hepatitis B, chronic hepatitis C, and chronic alcoholic liver disease [2, 3]. The treatment and prevalence of chronic liver disease vary widely from one type to another. For example, reports from the World Health Organization indicate that more than 90% of hepatitis C can be completely cured within 3–6 months [1]. In addition, there are various degrees of severity of chronic liver disease, such as chronic migratory hepatitis, slow-acting hepatitis, cirrhosis, and liver cancer. For each type and severity of chronic liver disease, the clinical outcomes, treatment drugs, and medical behaviors such as efficacy vary. Finding the cause of chronic liver disease is also very important for medical treatment [4]. The mechanisms of chronic liver disease are uncertain and complex and vary widely among individual patients. To address this situation, individualized treatment for different patients is needed to improve their therapeutic outcome [5]. It is thus clear that rapid prediction and accurate diagnosis of chronic liver disease are essential for the treatment of patients.

Chronic liver disease (CLD) is a global public health problem [1], and its causes include non-alcoholic fatty liver disease (NAFLD), chronic viral hepatitis, alcohol abuse, and autoimmune liver disease [2]. The early pathological changes of CLD are liver fibrosis, and when progressing to cirrhosis, life-threatening complications such as portal hypertension (PHTN) and hepatocellular carcinoma (HCC) can occur [3]. With the elimination of the underlying causes, liver fibrosis is expected to be reversed [4]. Early detection of fibrosis and its associated etiology is crucial. Liver biopsy is the gold standard for the assessment of liver fibrosis; however, there are drawbacks such as invasiveness and sampling errors.

In the process of personalized treatment of chronic liver disease, patients often need to check information on up to 80 tests related to them such as platelets, total bilirubin, alanine aminotransferase, creatinine, and so on. Among these kinds of information, how to quickly pinpoint which indicators are crucial to the cause of the patient's disease according to the individual characteristics of the patient is the key to the hospital's ability to prescribe the right medicine.

In this paper, we have proposed a modified BP neural network-based prediction model with improved ant colony optimization algorithm to process multiple index attribute items which are used to describe chronic liver disease. Additionally, the proposed model has the capacity to construct a chronic liver disease assessment model. Principal component analysis is used to explore and evaluate the impact of severity of patient's disease on each test index, which greatly reduces the dimensionality without losing majority of information. The dimensionality-reduced data were fed into an artificial neural network for training and used to diagnose and intelligently predict chronic liver disease, thus constructing an intelligent prediction model for chronic liver disease, which provides very important technical support for the treatment of chronic liver disease in hospitals.

The remaining sections of this paper are organized as follows.

In the subsequent section, various datasets utilized in the proposed BP neural network and ACO-based model were described in detail. In Section 3, background of the proposed model, that is, BP neural network and ACO, is described, whereas in the subsequent section, design and implementation guidelines of the proposed model are presented. Experimental results are presented in Section 5 which is followed by concluding remarks and future directions.

## 2. Benchmark Dataset

### 2.1. Data Source

Initially, 31 patients who were admitted to the Third Xiangya Hospital, specifically from March 2008 to May 2016, were selected, and the selection criteria were as follows:

1. All patients were diagnosed with chronic liver disease of different severity at a later stage.
2. All patients received routine blood, liver function, kidney function, and coagulation function tests. In this paper, the test data items of patients with different conditions and disease courses were considered as independent samples.

### 2.2. Generation of Dataset

Based on the patient data provided by the Third Xiangya Hospital, required test data and diagnostic results as well as the patients' basic information were imported into the database, and a total of 125 groups of 20-dimensional test indices related to chronic liver disease were initially selected as the research samples for this study. Among these values, 20-dimensional test indices are as follows.

1. Blood count: white blood cells (WBC), hemoglobin (Hb), platelets (PLT), and red blood cells (RBC).
2. Liver function: total bilirubin (TBIL), direct bilirubin (DBIL), alanine aminotransferase (ALT), aspartate aminotransferase (AST), total protein (TP), albumin (ALB), globulin (GLO), albumin-to-globulin ratio (A/G), and total bile acid (TBA).
3. Renal function: urea (UREA), creatinine (Cr), and uric acid (UA).
4. Coagulation: prothrombin time (TT), prothrombin time (PT), and prothrombin international normalized ratio (or international normalized ratio) (INR).
5. Basic information: age (AGE) and diagnostic result.

### 2.3. Preprocessing of Data

#### 2.3.1. Data Organization

In this study, results of each test index are kept in two decimal places and the descriptive words in the test data, such as “rechecked” and “verified,” are deleted. In medicine, “international normalized ratio (INR) of prothrombin” and “international normalized ratio” are the same index, which will be named as “international normalized ratio (INR) of prothrombin“ in this paper.

#### 2.3.2. Quantification of Diagnostic Results

The diagnostic outcomes were quantified into 4 categories based on the three-step progression of chronic liver disease from hepatitis, cirrhosis to liver cancer. To better match and distinguish between the predicted and expected groups, vectors were used to represent the quantified results. “000” denotes non-chronic liver disease; “001” denotes hepatitis; “010” denotes cirrhosis; and “100” indicates malignancy and liver cancer. Therefore, “0” represents non-chronic liver disease and “1” represents chronic liver disease. The specific quantitative results are listed in Table 1.

#### 2.3.3. Preferred Indicators

The ROC curve is a graph based on a series of two different subcategories (or thresholds) with the true positive rate (sensitivity) as the vertical coordinate and the false positive rate (1−specificity) as the horizontal coordinate. The area under the curve (AUC) was calculated from the ROC curve, and for AUC >0.5, the closer the AUC was to 1, the better the diagnosis was. In this experiment, 8 cases of non-chronic liver disease and 117 cases of chronic liver disease were diagnosed in 125 study samples.

## 3. Background of the Proposed Model

### 3.1. BP Neural Network Fundamentals

A BP neural network consists of an input layer, an implicit layer, and an output layer [6]. It is capable of approximating non-linear mappings with arbitrary accuracy and is a learning process based on signal propagation, where the signal is propagated in two processes: forward and backward propagation. Repeating its process, if the output value is close to the desired value, the training ends.

### 3.2. Basic Principles of Ant Colony Algorithm

Ant colony algorithm (ACA) [7, 8] is a search optimization algorithm that simulates an ant colony to find the optimal path from the nest to the food source. The pheromones released by ants during foraging have a communication function. The regulating effect of the positive feedback mechanism formed by the accumulation of pheromones speeds up the system to find the optimal solution and makes the ant foraging path proceed in the direction of the global optimum, thus obtaining the global relative optimal solution. In addition, the algorithm uses distributed parallel computing to perform a global search for the solution of the problem, avoiding the local minimal value problem.

### 3.3. Basic Principle of Combining Ant Colony Algorithm with BP Neural Network

BP neural network randomly generates initial weights and thresholds; if the initial values are not selected properly, the network will converge slowly or not or get a local minimum solution instead of a global optimal solution. BP neural network uses the gradient descent method to modify the weights and thresholds of the network to seek the optimal solution, so oscillation, network performance degradation, slow learning speed, falling into local minima, and other problems will occur. The ant colony algorithm has the advantages of intelligent global search optimization capability and better robustness. By training the weights and thresholds of BP neural networks with the ant colony algorithm, the non-linear mapping ability of BP neural networks and the global optimization ability of the ant colony algorithm can be combined to overcome the shortcomings of BP neural networks.

## 4. Design of Proposed Ant Colony and BP Neural Networks

### 4.1. Creation of New Transfer Function

The role of the transfer function in BP neural networks is to simulate the non-linear transfer characteristics of biological neurons, and the improper selection of the transfer function may lead to slow convergence, local minima, and other problems. In this paper, a new transfer function—Sch function—is established as

(1) $$\begin{array}{c} f\left(x\right)=\frac{2}{{\text{e}}^{x}+{\text{e}}^{-x}}. \end{array}$$

(*x*) has steeper and wider peaks near the origin of the coordinates, which can map the inputs of (−*∞*, +*∞*) into (0, 1), respectively. Since the liver function has no negative values and the information distribution is stored in the transfer function of each neuron, the Sch transfer function has better non-linear mapping capability than the conventional function in the BP neural network when the number of neurons is constant and enhances the massively parallel information processing capability. Since the topology of the network does not change, when the network computes the output value and the expected value close to each other, a large number of additional operations are not required, making the operation speed up.

### 4.2. Network Structure Optimization Determination

Although the data of liver function are non-stationary, the curve as a whole shows a normal distribution. The network structure chosen in this paper consists of 3 layers, and a prediction model that can accommodate large sample data is established:

(2) $$\begin{array}{c} y\left(t\right)=f\left\{\sum_{t=1}^{T}\omega_{jk}\left[f\left(\sum_{t=1}^{T}\omega_{ij}x_{i}-q_{j}\right)-q_{k}\right]\right\}\;t=1,2,\cdots ,T, \end{array}$$

where *y*(*t*) is the output value of the *t*th node of the network; *ω*_*ij*_ and *ω*_*jk*_ are the connection weights from the network output layer to the hidden layer and the connection weights from the hidden layer to the output layer; *q*_*j*_ and *q*_*k*_ are the thresholds from the network output layer to the hidden layer and from the hidden layer to the output layer, respectively; and *T* is the number of Sch functions, which are determined optimally by the minimum mean square error energy function. The minimum mean square error formula is

(3) $$\begin{array}{c} E_{\text{T}}=\frac{1}{2}\sum_{t=1}^{T}{\left[y\left(t\right)-y^{*}\left(t\right)\right]}^{2}, \end{array}$$

where *y*^*∗*^(*t*) is the measured value of liver function and *T* is determined using the stepwise test method. Given a value of fitting error *H* before prediction, if the minimum mean square error is less than *H*, *T* takes the value 1 and the value of *t* is calculated. If *t* < *H*, then *T* = 1; the optimal number is the hidden layers. The structure of the ant colony improved BP neural network in this paper is shown in Figure 1.

### 4.3. Ant Colony Algorithm for Improving BP Neural Network

If there are *n* weights and thresholds in the identified BP neural network structure, the weights and thresholds are numbered as *ω*_1_, *ω*_2_,...,*ω*_*n*_, and *ω*_*i*_ (1 ≤ *i* ≤ *n*) are set to *m* non-zero random values to form the set *Lω*_*i*_ (1 ≤ *i* ≤ *n*). If *Z* ants in the colony leave the colony to look for food, the pheromone of the *j*th element in the set will be the pheromone of the *j*th element. Each ant chooses one element from the set according to its information state and adjusts the pheromone of this element. The pheromone is calculated as

(4) $$\begin{array}{c} \tau_{j}\left(L_{\omega i}\right)\left(t+m\right)=\rho \tau_{j}\left(L_{\omega i}\right)\left(t\right)+\Delta \tau_{j}\left(L_{\omega i}\right),\\ \Delta \tau_{j}\left(L_{\omega i}\right)=\sum_{k=1}^{N}\Delta \tau_{j}^{k}\left(L_{\omega i}\right), \end{array}$$

where *ρ* is the persistence of residual information; *τ*_*j*_^*k*^(*L*_*ωi*_) is the pheromone left by the *k*th ant on the *j*th element of the set *L*_*ωi*_ in one cycle; and (*L*_*ωi*_)(*t*+*m*) is the pheromone on the *j*th element of the set *L*_*ωi*_ at the time of *t*+*m*.

It follows that the pheromone state transfer probability of the *k*th ant choosing the *j*th element on set *L*_*ωi*_ is

(5) $$\begin{array}{c} P\left[\sum_{k=1}^{N}\Delta \tau_{j}^{k}\left(L_{\omega i}\right)\right]=\frac{\tau_{j}\left(L_{\omega i}\right)}{\sum_{k=1}^{N}\Delta \tau_{j}^{k}\left(L_{\omega i}\right)}. \end{array}$$

The selection of a set of weights and thresholds in the BP neural network is completed when all *Z* ants in *L*_*ωi*_ have selected an element to reach the food source. Then, the ants return to the anthill in the same way, while optimally adjusting the pheromones of the elements selected by the ants and finding the global optimal solution during repeated iterations. The flow of the ant colony improved BP neural network algorithm in this paper is shown in Figure 2.

## 5. Experimental Setup and Results

### 5.1. Comparative Analysis of Predicted Effects

Under the condition that the topology and parameters of the BP nerve network remain unchanged, samples A (the streamlined sample set after ROC preference and dimensionality reduction by principal component analysis) and B (the original 20-dimensional sample set) are used as input to construct an intelligent prediction model to validate the test samples.

In order to better and more objectively evaluate the prediction accuracy of both A and B, the experiment will be repeated 1000 times, and the training samples will be randomly selected in each experiment, and the average of all the results will be taken as the final prediction accuracy.  Figure 3 shows the accuracy of the hidden layer nodes of 8, 11, 14, and 17, respectively, using the data before and after dimensionality reduction as the input of the BP neural network.

Figure 4 shows the convergence of the BP neural network for sample set A after dimensionality reduction using ROC preference and principal component analysis, where the horizontal coordinate is the number of iterations, the vertical coordinate is the mean square error, and the dashed line is the optimal mean square error reference line.  Figure 5 shows the convergence of the BP neural network with 20-dimensional original dataset B as input under the same conditions. Comparing Figures 4 and 5, it is easy to conclude that A converges faster than B.

### 5.2. Algorithm Verification

In this study, historical liver function and patient information were provided by our hospital. Complete liver function, specifically from July 1, 2012, to August 1, 2014, was similar and variation of factors such as blood routine, kidney function, and coagulation function was also very small, and this paper used a classification method by month for liver function prediction, with 12 prediction models. This classification method greatly reduces the amount of operations and redundancy of information and improves the training speed. The models predicted liver function on November 25, 2013, January 31, 2014, April 17, 2014, and July 2, 2014, respectively, with a prediction time scale of 15 min. The prediction results are shown in Figure 6.

Figure 6(a) shows the measured and predicted liver function on November 25, 2013. Historical liver function, blood routine, kidney function, and coagulation function for November 2012 and November 1–24, 2013, were used as inputs to the January model, with 1,620 historical liver function data and a total of 486 factors affecting liver function, for a total of 1,620 data were trained on the neural network. For the prediction of liver function on November 25, 2013, after repeated training, the ant colony parameters were chosen as follows: *ρ* = 0.7, the number of ants was 32, the information intensity was 54, and the optimal number of hidden layers was 10. As shown in Figure 6(a), the predicted values match with the measured values, and the prediction is good.  Figure 6(b) shows the measured and predicted values of liver function on January 31, 2014. A total of 1,654 data of historical liver function and influencing factors were used as input to train the January neural network, and after repeated training, the ant colony parameter was chosen as *ρ* = 0.6, the number of ants was 32, the information intensity was 41, and the optimal number of implied layers was 11, and the prediction achieved good results.  Figure 6(b) also shows the measured and predicted values of liver function on January 31, 2014. The blood routine, kidney function, and coagulation function on that day were cloudy/overcast, the maximum temperature was 15°C, the minimum temperature was 8°C, the air quality index was 67, the average wind speed was 1.774 57 m/s, the average relative humidity was 31.907 21%, the sunshine hours were 12.75 h, and the atmospheric pressure was 93.48 kPa, putting a total of 2,817 data on historical liver functions, and influencing factors were used as input to train the neural network, and the ant colony parameter was chosen as *ρ* = 0.8, the number of ants was 51, the information intensity was 76, and the optimal number of hidden layers was 10.

The above prediction results show that the prediction method by month is reasonable, and the prediction results under different blood routine, renal function, and coagulation function types have good prediction accuracy. The error of individual prediction points is larger, which may be because the measured data contain some bad points due to the measurement instrument error factor in the data collection, and the randomness and uncertainty of blood routine, kidney function, and coagulation function types make the prediction results inaccurate. But overall the predicted value is close to the actual measured value.

### 5.3. Comparison with RMSE of BP Neural Network Model

To estimate the prediction model results, the proposed model uses root mean square error (RMSE), which is

(6) $$\begin{array}{c} \text{RMSE}=\sqrt{\frac{\sum_{i=1}^{n}{\left(y-y^{*}\right)}^{2}}{n}}, \end{array}$$

where *n* is the number of outputs of the network.

The prediction results of liver function based on the ant colony improved BP neural network model were compared with the prediction results of BP neural network model for the above four days, which showed that the ant colony improved BP neural network model effectively improved the prediction accuracy of special blood routine, kidney function, and coagulation function types. The RMSE comparison results are shown in Table 2.

## 6. Conclusion and Future Work

In this paper, we propose a modified BP neural network with improved ant colony algorithm to process multiple index attribute items describing chronic liver disease to construct a chronic liver disease assessment model. Experiments show that the proposed model not only reduces the complexity but also improves the prediction accuracy by 15.07%. In large-scale high-dimensional incremental learning samples, the algorithm not only ensures the classification accuracy and good generalization ability but also the learning training speed is faster than the classical SVM incremental learning algorithm, which can perform incremental learning quickly.

In the future, with the continuous improvement of MRE imaging technology, we will be able to quantify the microscopic characteristics of different chronic liver diseases such as hepatocyte fat content, iron deposition, and viscoelasticity in a non-invasive, accurate, reproducible, and precise manner, thus providing an opportunity for early detection and follow-up assessment of chronic liver diseases and providing a reference for the development of individualized treatment strategies for patients.

## Figures and Tables

**Figure 1:** Ant colony improved BP neural network structure.

**Figure 2:** Flow of ant colony improved BP neural network algorithm.

**Figure 3:** Accuracy comparison before and after dimensionality reduction.

**Figure 4:** Convergence speed of A sample set when number of nodes in the hidden layer is 17.

**Figure 5:** Convergence speed of B sample set when number of nodes in hidden layer is 17 and training speed of overall incremental learning.

**Figure 6:** Prediction result curve. (a) Forecast result curve for January 25, 2013. (b) Forecast result curve as of January 31, 2014.

**Table 1:** Quantification results.

Diagnostic results	Quantized value	Vector	Explanation
Parson's disease (PD), gallstones	0	000	Non-chronic liver disease
Hepatitis		001	Hepatitis
Viral hepatitis cirrhosis			
Alcoholic cirrhosis	1	010	Cirrhosis
Liver mass, liver cancer			
PLC (primary liver cancer)		100	Liver cancer

**Table 2:** RMSE comparison results.

Prediction model	Sunny	Sunny/cloudy	Cloudy/cloudy	Cloudy/thunderstorm
Ant colony BP model	8.4317	9.7340	12.7375	13.651814.6527
BP model	14.6527	17.6298	29.4519	38.7219

## Data Availability

The datasets used and analyzed during the current study are available from the corresponding author upon reasonable request.
